The article "Smart Healthcare System for Severity Prediction and Critical Tasks Management of COVID-19 Patients in IoT-Fog Computing Environments" was retracted in 2023. Reasons: signs of a paper mill; suspected computer-generated content; unreliable results or conclusions; lack of ethics approval or compliance.

# Smart Healthcare System for Severity Prediction and Critical Tasks Management of COVID-19 Patients in IoT-Fog Computing Environments

**DOI:** 10.1155/2022/5012962

**Published:** 2022-07-19

**Authors:** Karrar Hameed Abdulkareem, Ammar Awad Mutlag, Ahmed Musa Dinar, Jaroslav Frnda, Mazin Abed Mohammed, Fawzi Hasan Zayr, Abdullah Lakhan, Seifedine Kadry, Hasan Ali Khattak, Jan Nedoma

**Affiliations:** ^1^College of Agriculture, Al-Muthanna University, Samawah 66001, Iraq; ^2^College of Engineering, University of Warith Al-Anbiyaa, Karbala, Iraq; ^3^Ministry of Education, General Directorate of Curricula, Pure Science Department, Baghdad, Iraq; ^4^Engineering Department, University of Technology- Iraq, Baghdad, Iraq; ^5^Department of Quantitative Methods and Economic Informatics, Faculty of Operation and Economics of Transport and Communication, University of Žilina, Žilina, Slovakia; ^6^Department of Telecommunications, Faculty of Electrical Engineering and Computer Science, VSB-Technical University of Ostrava, Ostrava, Poruba, Czech Republic; ^7^College of Computer Science and Information Technology, University of Anbar, 11, Ramadi, Anbar, Iraq; ^8^Department of Biochemistry, College of Medicine, University of Wasit, Wasit, Iraq; ^9^Department of Computer Science and Artificial Intelligence, Wenzhou University, Wenzhou 325035, China; ^10^Noroff University College, Kristiansand, Norway; ^11^School of Electrical Engineering and Computer Science, National University of Sciences and Technology (NUST), Islamabad 44500, Pakistan

## Abstract

COVID-19 has depleted healthcare systems around the world. Extreme conditions must be defined as soon as possible so that services and treatment can be deployed and intensified. Many biomarkers are being investigated in order to track the patient's condition. Unfortunately, this may interfere with the symptoms of other diseases, making it more difficult for a specialist to diagnose or predict the severity level of the case. This research develops a Smart Healthcare System for Severity Prediction and Critical Tasks Management (SHSSP-CTM) for COVID-19 patients. On the one hand, a machine learning (ML) model is projected to predict the severity of COVID-19 disease. On the other hand, a multi-agent system is proposed to prioritize patients according to the seriousness of the COVID-19 condition and then provide complete network management from the edge to the cloud. Clinical data, including Internet of Medical Things (IoMT) sensors and Electronic Health Record (EHR) data of 78 patients from one hospital in the Wasit Governorate, Iraq, were used in this study. Different data sources are fused to generate new feature pattern. Also, data mining techniques such as normalization and feature selection are applied. Two models, specifically logistic regression (LR) and random forest (RF), are used as baseline severity predictive models. A multi-agent algorithm (MAA), consisting of a personal agent (PA) and fog node agent (FNA), is used to control the prioritization process of COVID-19 patients. The highest prediction result is achieved based on data fusion and selected features, where all examined classifiers observe a significant increase in accuracy. Furthermore, compared with state-of-the-art methods, the RF model showed a high and balanced prediction performance with 86% accuracy, 85.7% F-score, 87.2% precision, and 86% recall. In addition, as compared to the cloud, the MAA showed very significant performance where the resource usage was 66% in the proposed model and 34% in the traditional cloud, the delay was 19% in the proposed model and 81% in the cloud, and the consumed energy was 31% in proposed model and 69% in the cloud. The findings of this study will allow for the early detection of three severity cases, lowering mortality rates.

The article "Smart Healthcare System for Severity Prediction and Critical Tasks Management of COVID-19 Patients in IoT-Fog Computing Environments" was retracted in 2023. Reasons: signs of a paper mill; suspected computer-generated content; unreliable results or conclusions; lack of ethics approval or compliance.

## 1. Introduction

COVID-19 has a destructive impact on people's lives and healthcare services all around the globe [1]. Therefore, it is essential to diagnose affected patients as soon as possible to prevent the spread of the COVID-19 [2]. As a result, the rising incidence of COVID-19 presents another threat to the health field, in addition to the projected daily service rendered, in which mortality is assumed to be high, and diagnosis takes a long time [3]. Countries' experiences during the initial wave of the pandemic revealed the disease's vulnerability to healthcare systems [4]. Additionally, the rapid global spread of the COVID-19 pandemic is imposing high pressure on the entire human society. Furthermore, COVID-19 impacts work-related processes, placing strain upon many employees in project teams. Identifying process variables and potential organizational resources can play an essential role in addressing employee mental health, both for the current pandemic and future crises [5]. Thus, the prevention and control of future global health emergencies must be a priority [6]. Since the COVID-19 epidemic has become a pandemic, it would be critical to have resources to quickly classify people at the most significant risk of mortality and morbidity. In addition, infections also lead to nosocomial spread, which has an effect on healthcare staff and the overall delivery of treatment [7].

Due to the popularity of machine learning (ML) models in the diagnosis of different diseases [8], these models could be able to provide an accurate and efficient COVID-19 solution that aids in the early detection of disease [9, 10]. Machine learning has been widely used to reduce the healthcare systems burden [11]. Furthermore, it has the potential to reduce the decision time linked with conventional methods of detection [12]. The advancement of the estimation, reduction, and monitoring of potential global health threats is considered a crucial factor in the growth of AI strategies to identify the risks of infectious diseases [13]. Several researchers have published on various forms of AI classifiers using actual COVID-19 datasets with various case studies and goals [14]. Earlier researches have concentrated on mortality predictions [15], diagnosis [2], severity valuation, and illness progression [16]. Most present methods have utilized ML methods for prediction based on medical images [17] and other clinical markers [3]. Most machine learning approaches have been utilized to predict and diagnose COVID-19, while fewer studies have focused on severity prediction.

The article "Smart Healthcare System for Severity Prediction and Critical Tasks Management of COVID-19 Patients in IoT-Fog Computing Environments" was retracted in 2023. Reasons: signs of a paper mill; suspected computer-generated content; unreliable results or conclusions; lack of ethics approval or compliance.

Taking into consideration the multiple complications involved with COVID-19 [18], approaches that can triage COVID-19 patients may assist in prioritizing treatment for those at a high risk of serious illness. COVID-19 severity may be classified as the following: ordinary, mild, critical, and severe [19]. Severe cases necessitate more medical attention and energy than minor and routine cases. A high rate of false-positive severe or vital cases might cause healthcare services to become overburdened (i.e., beds in the intensive care unit). Furthermore, delays in reporting severe or urgent cases would result in patients with a greater risk of death receiving delayed care. As a result, identifying acute conditions as soon as possible is critical so that services may be deployed and care may be intensified [20].

According to Reference [21], a method is needed for real-time processing of COVID-19 patient data with ultra-low latency, prediction of COVID-19 infection at an early stage, and generation of an emergency warning and medical records for the person, their guardian, and doctors/experts. In this case, IoT cloud/fog computing combined with machine learning could be the most effective solution [22]. Numerous healthcare institutions are implementing cloud/fog computing in healthcare to achieve optimum effectiveness in the fight against different diseases. At the same time, machine learning can help classify a user's health status at an early stage [23]. Because of the adequate storage and simplicity of processing large volumes of medical data at a low cost, cloud computing is the most efficient and appropriate tool for improving the efficiency of healthcare services [24].

The article "Smart Healthcare System for Severity Prediction and Critical Tasks Management of COVID-19 Patients in IoT-Fog Computing Environments" was retracted in 2023. Reasons: signs of a paper mill; suspected computer-generated content; unreliable results or conclusions; lack of ethics approval or compliance.

Fog computing offers a real-time approach with minimal latency [25]. As a result, fog computing may improve application service delivery time while reducing network congestion. On the one hand, the existing fog computing architecture does not support dispersed network architecture. The fault and load results of the fog node are therefore displayed [26]. On the other hand, existing fog computing architecture does not support dispersed network architecture. So, effective management of applications is crucial to use the capabilities of fog nodes [25]. As a result, combining cloud-fog innovations could result in a world-record-breaking approach for the healthcare industry [27]. A gateway node acts as a point of access to the remaining system. The gateway collects the sensed data from the connected sensors. The standard computing system operating many applications may be efficiently used with the agents distributed through the system that separately function for the users. The agents coordinate the communities and cooperate in providing intelligent and customized services depending on different users' contexts [28]. Multi-agent systems (MASs) have been widely used to solve real-world problems because they are proactive and flexible to environmental changes. The authors of [29] suggest a home hospitalization system for COVID-19 based on cloud computing, fog computing, and the Internet of Things (IoT), which are three of the essential technologies that have significantly aided the growth of the healthcare sector. The suggested environmental sensing unit consists of three modules (smoke, gas, humidity, and temperature) for environmental component detection.

However, detecting the signs mentioned above will exhaust the network because the detected signs have no impact on the detection of COVID-19 infection. To prevent COVID-19 and future pandemics, the authors of [30] describe a cooperative multi-agent robot system (MARS) for strictly enforcing physical distancing restrictions in broad areas using human-robot interaction (HRI). The authors employed multiple self-docking autonomous robots with collision-free navigation to enforce physical distancing limitations by delivering alert signals to those who did not comply. However, this paper employs a multi-agent system for monitoring the distance without any effort to predict COVID-19 infection.

The main contributions of our study can summarize into following list:

- Propose a Smart Healthcare System for Severity Prediction and Critical Tasks Management (SHSSP-CTM) of COVID-19 patients in IoT-Fog computing.
- Propose a fusion process in order to find the best combination of COVID-19 patient characteristics such as demographic, chronic conditions, symptoms, and laboratory findings that interpreted the importance of distinct feature set with the highest predictive power.
- Present COVID-19 severity prediction model with sufficient predictive power based on the balanced dataset, fusion process, and feature selection method.

The article "Smart Healthcare System for Severity Prediction and Critical Tasks Management of COVID-19 Patients in IoT-Fog Computing Environments" was retracted in 2023. Reasons: signs of a paper mill; suspected computer-generated content; unreliable results or conclusions; lack of ethics approval or compliance.

The rest of this study is as follows: related work on Smart Healthcare System for Severity Prediction and Critical Tasks Management of COVID-19 patients is given in Section 2. Clinical, laboratory, vital functions, and medical history information are collected from hospital records in Section 3. In Section 4, the description of the methods of the Smart Healthcare System for Severity Prediction and Critical Tasks Management of COVID-19 patients is provided. The analysed results of the proposed system via different techniques with different methods are presented in Sections 5 and 6.  Section 7 introduced a comparison based on different state-of-the-art studies.  Section 8 highlighted the constraints in the proposed study. Finally, Section 9 concludes the research conclusion and future work.

## 2. Related Works

Meanwhile, several organizations looked at ways to categorize cases based on severity using ratings and rating schemes to aid clinicians in the diagnosis and triage [31]. The COVID-GRAM score was developed by Lian et al. to predict acute disease in deceased patients admitted to an intensive care unit (ICU) or mechanically ventilated [32]. This score utilized ten variables, yielding an area under the curve (AUC) of 0.88 in their receiver operating characteristics (ROC) analysis. Based on data from 208 Chinese patients, Ji et al. created the CALL score (*C* = comorbidity, *A* = age, *L* = lymphocyte count, and *L* = lactate dehydrogenase) to assess disease progression. In their growth cohort, their model utilized four variables and returned an AUC of 0.91 [33]. Another score was suggested by an American group that used 641 patients to estimate intensive care entry or mortality. Their score predicted ICU entry with an AUC of 0.74 and death of 0.82 [34]. The CURB-65 (*C* = confusion, *U* = blood urea nitrogen, *R* = respiratory rate, and 65 = age 65 or older) score and the Pneumonia Severity Index (PSI) were both utilized on 681 laboratory-confirmed Turkish patients to estimate mortality of COVID-19-related pneumonia, with AUCs of 0.88 and 0.91, respectively [35]. The low AUC output has been shown for the whole of these scores, which were generated utilizing multivariate regression models.

In Reference [31], authors have made efforts to measure the predictive accuracy of the WHO COVID-19 severity classification on 295 COVID-19 admitted patients. The whole patients were categorized depending on WHO severity categorization at admission: moderate, severe, and critical. The good outcome of this study is that a Bayesian network analysis was utilized to generate a model for analysing the predictive accuracy of the WHO severity classification and generate the EPI SCORE. However, there is still room to improve classification performance with more variables and feature combinations. This study has scored only 83.8% and 91% as AUC scores for the models depending on WHO category only and our EPI SCORE, respectively. According to [7], other well-validated assessment tools for pneumonia seriousness did not work well. None of the patients who experienced acute respiratory distress syndrome (ARDS) may have fulfilled the pneumonia medical outcomes testing team (PORT) score's requirements for requiring hospitalization. Instead, it was discovered that a mixture of factors widely obtained at the time of initial presentation could forecast illness progression to ARDS. Combining more COVID-19 characteristics provides a more complete and more accurate prediction performance [20].

The article "Smart Healthcare System for Severity Prediction and Critical Tasks Management of COVID-19 Patients in IoT-Fog Computing Environments" was retracted in 2023. Reasons: signs of a paper mill; suspected computer-generated content; unreliable results or conclusions; lack of ethics approval or compliance.

The authors in Reference [7] display a first step toward creating an artificial intelligence (AI) system through algorithmically identifying the COVID-19 clinical features, which forecast outcomes, then improving a method for predicting patients at risk for the more serious disease at the time of initial presentation. However, this study has scored low prediction performance where the predictive models learned from patients' empirical data from two hospitals forecasting extreme cases with an accuracy of 70% to 80%. Based on a combination of clinical and imaging results, the authors in [20] established a machine learning method for automatic COVID-19 severity assessment. Imaging features had the most significant influence on model production, and a mix of imaging and clinical features produced the optimum overall results. The main classification task was based on recognizing the difference between severe and mild cases. This research demonstrated that imaging and clinical tools might be utilized to simplify COVID-19 severity assessment, better triage COVID-19 patients, and optimize treatment for those at a greater risk of severe disease. However, since the data collection was heavily skewed, models may have been overfit to the majority class. Furthermore, since this analysis only used patient baseline results, it could not determine how early COVID-19 development can be identified. Another issue that could be presented, especially when with imaging features, is that considering their benefits, medical images of COVID-19, and other forms of pneumonia may share specific similar imagery characteristics, making automatic differentiation challenging [36, 37]. This study has scored high prediction results with 95% as the AUC value. However, low prediction can be seen where only 60% scored as F-measure and 76% as precision value, respectively. However, all previous works have considered the severity prediction for COVID-19 and ignored the importance of task scheduling for the critical case that may result in death if no mechanism is adopted.

The article "Smart Healthcare System for Severity Prediction and Critical Tasks Management of COVID-19 Patients in IoT-Fog Computing Environments" was retracted in 2023. Reasons: signs of a paper mill; suspected computer-generated content; unreliable results or conclusions; lack of ethics approval or compliance.

## 3. Dataset

Samples were collected between 4/8/2020 and 3/12/2020 and were used for model development. The total number was 78 people infected with the COVID-19 virus, diagnosed under the supervision of specialized doctors at Al Aziziya Primary Healthcare Sector, Wasit Governorate, Iraq. For 78 patients, they lost sense of taste and smell, which was the most common symptoms (92.3% and 91.02, respectively) and followed by fever (67.95%), generalized weaknesses (66.67%), cough (58.97%), sore throat (57.69%), sneezing (56.41%), pleuritic chest pain (53.84%), diarrhoea (52.56%), and nasal congestion and rhinorrhoea (42.30%) as shown in Table 1.

## 4. Smart Healthcare System for Severity Prediction and Critical Tasks Management of COVID-19 Patients

Recently, smart healthcare systems considered to be a developing application of the Internet of Medical things (IoMT). The smart healthcare framework comprises of wearable sensors utilized to monitoring the particular health status of the patients or users. Most critically, wearable innovation has become a crucial role of not just remote patients monitoring but moreover for users health monitoring frequently. The wearable devices can help in minimizing the visit of specialists or doctors in health monitoring.

It moreover helps within the early identification of smart hospital development, diseases, safety provisioning, and drug research. The two main innovations need to be explored to enhance a smart healthcare framework. Firstly, through biomedical sensors like blood pressure, patient priority, temperature, motion, and how the wearable devices are appended on the users body to acquire, their health status is studied. As shown in Figure 1, the framework of the suggested smart healthcare system is discussed in this section. The SHSSP-CTM has two chief data sources. The first one appeared on the left and is the Internet of Medical Things (IoMT) sensor data. The second data source is Electronic Health Records (EHRs).

An agent will run in each gateway, and it is role forwarding stream sensed data of each patient through Wi-Fi and Bluetooth to fog layer. The purpose of the COVID-19 severity prediction model is predicting the risk disease for patients depending on the gathered information. This engine contains of four major steps: (1) information fusion; (2) preprocessing; (3) ML model depending on COVID-19 severity forecast. The extracted features from unstructured and structured information are fused in the first stage, utilizing the suggested fusion scheme. The information is then preprocessed utilizing information mining approaches in the next step. Data normalization and useful feature selection approaches are included in this step. For the final prediction of patient severity, the preprocessed information is transferred to an ML classifier trained on a COVID-19 dataset in the third stage. After data preprocessing and prediction with diagnosis steps, (4) multi-agent system will assign (prioritize) the tasks according to criticality. Patient with sever criticality will be assigned to ICU. Patient with moderate criticality will be advised to be in continuous monitoring. In last case, when the patient is in mild criticality, this will be advised for further checking. Two main tasks are handled by cloud datacentres: first task is processing the stream sensed tasks when all fog nodes are busy and no available resources, and second task is upgrading patients' history records.

The article "Smart Healthcare System for Severity Prediction and Critical Tasks Management of COVID-19 Patients in IoT-Fog Computing Environments" was retracted in 2023. Reasons: signs of a paper mill; suspected computer-generated content; unreliable results or conclusions; lack of ethics approval or compliance.

### 4.1. Multisource COVID-19 Data Collection

The proposed SHSSP-CTM for COVID-19 patients considers several sorts of information for severity prediction of COVID-19 such as Internet of Medical Things (IoMT) sensors, and Electronic Health Record (EHR) data as displayed in Figure 1. The first type of information is gathered with wearable sensors help. The IoMT sensors data include body temperature and saturation of oxygen in the blood (SPO_2_). These IoMT sensors' data offer valued data for the severity prediction and management of critical COVID-19 patient. All IoMT sensor information is allocated in the information collection layer (e.g., S1 is SPO_2_ sensor data). During processing, the system finds those identities to be features. Additionally, for further processing, the IoMT sensor information is displayed in columns, along with identities and numerical values. Furthermore, shapeless EHRs of the patient are gathered to more sever issues for COVID-19 patient.

EHRs include demographic, chronic conditions, symptoms, and laboratory findings data. The EHRs may be examined for extracting valued data, which may assist in severity management and prediction of critical COVID-19 patient. Each of demographic, chronic conditions, symptoms, laboratory findings, and vital sign feature set will be used as first input in the COVID-19 severity prediction phase.

The article "Smart Healthcare System for Severity Prediction and Critical Tasks Management of COVID-19 Patients in IoT-Fog Computing Environments" was retracted in 2023. Reasons: signs of a paper mill; suspected computer-generated content; unreliable results or conclusions; lack of ethics approval or compliance.

### 4.2. COVID-19 Severity Prediction

This layer will be as cornerstone for indicating severity prediction. Also, this layer clarifies the suggested ML severity prediction model that is composed of two major processes, feature extraction and severity prediction process, as displayed in Figure 2. However, all processes in this layer and next layers will be executed based on the proposed dataset.

#### 4.2.1. Feature Extraction

The related data obtained from raw information are significant in COVID-19 severity prediction because of its direct effect on prediction performance. The major source for feature extraction process is mainly EHR and IoMT sensors' data that are main indicators for severity of COVID-19 patient. Also, the extracted features are in different data forms such as numerical and categorical. In numerical features, the system obtains factors in which values are already obtainable in an organized form. As such, the system obtains feature with a different range of numbers, for example, age, body temperature, SPO_2_, creatinine, and other values from structured areas. In categorical feature extraction, the system derives risk factors with values that fall into various groups mainly between two values (zero or one) such as diabetes history, heart disease, male, female, and nasal congestion. To mention, this process will applied into three main scenarios based on number of features such as single feature set, feature fusion set, and feature selection with fusion set.

#### 4.2.2. ML Severity Prediction Model

The severity prediction process was performed on the base of the identified dataset, the employment of several ML models, and extracted features. Python was utilized for the whole forecast tasks through the study time. The last severity prediction model output for COVID-19 was produced in this subphase in which multiclass classification was performed. In other words, three cases that the ML models have to predicate specifically: mild, moderate, and sever cases. According to Reference [20], logistic regression (LR) can provide good prediction power for COVID-19 severity cases that is why used this technique as first baseline prediction model in this study. Furthermore, for more generalization process, we used also random forest (RF) as second baseline prediction model. In latest research, random forest was found to be more stable and resilient than extreme learning machines, neural networks, and SVMs, particularly with limited training sets [38]. However, in order to show prediction power of mentioned models three main scenarios are included in the prediction process such as prediction based on single feature set, prediction based on feature fusion set, and prediction based on feature selection with fusion set. However, the first input for this phase is five feature sets that predicted and extracted individually, which is explained as follows:

 
*Set 1*: demographic features such as age and gender.
 
*Set 2*: chronic condition features such as heart disease, diabetes, and cancer.
 
*Set 3*: symptoms features such as cough, fever, nasal congestion, generalized weakness, sneezing, rhinorrhoea, diarrhoea, pleuritic chest pain, sore throat, lost sense of smell, and lost sense of taste.
 
*Set 4*: laboratory finding features such as haemoglobin, platelet count, lymphocyte count, white blood cell count, C-reactive protein, urea, and creatinine.
 
*Set 5*: vital signs features such as SPO_2_ and body temperature.

The article "Smart Healthcare System for Severity Prediction and Critical Tasks Management of COVID-19 Patients in IoT-Fog Computing Environments" was retracted in 2023. Reasons: signs of a paper mill; suspected computer-generated content; unreliable results or conclusions; lack of ethics approval or compliance.

### 4.3. Multisource Feature Fusion

The fusion of EHR and IoMT sensor information is discussed in this section, as seen in Figure 2. Fusion is the process of combining data from various databases to provide more valuable and valid information for classification [39, 40]. Data function and decision levels are the three fusion levels [41–43]. Data-level integration brings together several datasets from disparate sources.

There are two types of data fusion: feature and decision levels. At the feature level, features are extracted one by one from various datasets and then combined to form the optimal selection of features for prediction [44]. Even though many studies proposed feature extraction of COVID-19 patient from medical images [45] or laboratory findings [46], the accuracy obtained from classification was not quite significant. Meanwhile, studies for COVID-19 prediction believe that the combination of more than one data or feature type for instance clinical and imaging features is decent to improve the prediction accuracy [7, 20]. Thus, fusion process is considered in this study in order to improve the system prediction accuracy.

Data-level fusion normally requires a vast volume of redundant information, making it undesirable. The feature level, on the other hand, provides enough data to determine the COVID-19 severity. Feature-level fusion is achieved in the suggested framework. Figure 2 depicts the function fusion workflow. First, sensors are used to capture the patient's physiological information, and EHR is retrieved, as discussed in the data collection layer, respectively. The data from IoMT sensors are then combined with information derived from EHR data. Lastly, the data from the IoMT sensor and the derived features are translated to comma separated value (CSV) files. As a result, the system determines the optimal mix of features connected to COVID-19 severity prediction. However, in this phase, five main feature sets that already mentioned in the previous phase are fused (*Set 1*, *Set 2*, *Set 3*, *Set 4*, and *Set 5*). Furthermore, the fusion process will formed a new feature vector that consist of 25 severity variables for COVID-19 patients form different data sources. The main goal of the proposed system is predicting COVID-19 patients' severity with relevant and lower-dimensional features extracted from multisource data.

The article "Smart Healthcare System for Severity Prediction and Critical Tasks Management of COVID-19 Patients in IoT-Fog Computing Environments" was retracted in 2023. Reasons: signs of a paper mill; suspected computer-generated content; unreliable results or conclusions; lack of ethics approval or compliance.

However, the derived features from IoMT sensor data can contain irrelevant data, lowering prediction accuracy, and increasing feature dimensionality. Furthermore, those also improve the memory requirements and classification complexity. As a result, data preprocessing is performed prior to actual processing, which increases data accuracy while still saving memory and time.

### 4.4. Data Preprocessing

Preprocessing information is the most important phase before using machine learning algorithms. Real-world information cannot be used explicitly in the prediction task because it is incomplete, noisy, and contradictory. As a result, a preprocessing stage is used to efficiently reflect the information for COVID-19 severity prediction. Normalization and feature selection are examples of data preprocessing in this study.

#### 4.4.1. Data Normalization

Before execute the feature selection approach, we have to deal with data from heterogeneous resource, so huge differences in the feature scales can be presented. The proposed dataset has a lot of features, and each feature has several numerical values that make the calculation process more complex. As a result, the dataset is normalized using a normalization process. Since each function has equal importance, normalization aims to make any data point, which has the same size [3]. The translation of the minimum value of every feature into 0 is the highest value into 1, and the other values have to be a decimal between 0 and 1. The formula for min-max normalization is as follows:

(1) $$\begin{array}{c} v{\;}^{\prime }=\frac{\left(v-\min\right)}{\left(\max-\min\right)}, \end{array}$$

where *v* ′ denotes for normalized data value, *V* represents original data value, min represents minimum data value, and max denotes for maximum data value.

#### 4.4.2. Feature Selection Based on Information Gain Method

Feature selection is essential step, especially after executed feature extraction process and tackling the issues of non-normalized data. In most cases, patient reports have a lot of useless information in them, which reduces the accuracy of forecast. Consequently, extracting useful data from medical records, minimizing noise through excluding irrelevant features, and accurately prediction with a small number of features are all difficult tasks. It is critical to eliminate noisy data, pick useful features that aid in reliable performance, and lessen the dataset's sophistication and dimensionality before implementing any prediction model. As a result, feature selection is an essential move which increases data clarity and reduces ML model training time. We employ the data gain approach, which has an impact on prediction performance by removing noisy functions. The standardized proposed dataset for COVID-19 intensity prediction has 25 attributes. Just a few of them are helpful in predicting the magnitude of a situation into one of the divisions. Depending on the relevance of features in the dataset, the system may learn about complex issues. Utilizing information gain (IG), the suggested system selects features, which quantify significance in relation to the classification task. The suggested system measures system instability using entropy. It calculates the difference between before and after entropy of two distinct variables, *A* and *B*, as seen in the equations below [47]:

(2) $$\begin{array}{c} IG\left(\frac{A}{B}\right)=H\left(A\right)-H\left(\frac{A}{B}\right). \end{array}$$

Equations (2) and (3) can be used to calculate the prior entropy of feature *A*, where *A* and *B* are discrete random variables:

(3) $$\begin{array}{c} H\left(A\right)=-\sum_{i}P\left(A_{i}\right)\log_{2}\;P\left(A_{i}\right), \end{array}$$

where *P* (*A*_*i*_) represents the prior probability. After being specified postentropy *B*, the conditional entropy of *A* may be computed using

(4) $$\begin{array}{c} H\left(\frac{A}{B}\right)=-\sum_{i}P\left(B_{j}\right)H\left(\frac{A}{B_{j}}\right)=-\sum_{i}P\left(B_{j}\right)\sum_{i}P\left(\frac{A_{i}}{B_{j}}\right)\log\;2\;P\left(\frac{A_{i}}{B_{j}}\right), \end{array}$$

(5) $$\begin{array}{c} IG\left(\frac{A}{B}\right)=-\sum_{i}P\left(A_{j}\right)\log_{2\;}\;P\left(A_{i}\right)-\left(\sum_{i}P\left(B_{j}\right)\sum_{i}\left(P\left(A_{i},B_{j}\right)\log\;2\;P\left(A_{ij}\right)\right)\right). \end{array}$$

Utilizing equation (5), the suggested scheme calculates the value of every attribute to the role of COVID-19 severity prediction. After calculating the IG for every feature, this method deletes the least relevant features. It removes features through removing one at a time before the decrease in performance stops.

The article "Smart Healthcare System for Severity Prediction and Critical Tasks Management of COVID-19 Patients in IoT-Fog Computing Environments" was retracted in 2023. Reasons: signs of a paper mill; suspected computer-generated content; unreliable results or conclusions; lack of ethics approval or compliance.

### 4.5. Critical COVID-19 Patient Management

#### 4.5.1. Multi-Agent Algorithm (MAA)

The study devises the MAA to handle the initial workload assignment in the fog cloud network. The workloads created through this application are variable length, dynamic, and need priority implementation at cloud and edge. In healthcare environment, applications fight for restricted resource devices. At different nodes of fog, those workloads are executed and allocated. If basic round-robin (RR) algorithm using the first-come-first-served (FCFS) method is utilized for job scheduling in computing fog, it provides equivalent priority to the whole tasks, resulting to increase time of response for tasks with limited burst times. However, the goal of computing fog paradigm is minimizing time of waiting, time of response, and traffic of network [17]. So, a task scheduling algorithm in fog needs for designing and implementing with the next goals, reduces the time spent in the loop of application (latency); uses the fog gadgets in a professional manner (RAM, processor, energy, etc.), and lessens the use of network.

In Step 1, personal agent analysed the all nodes and sort them according to their characteristics. Priority task scheduling (PTS) is based on the following characteristics: dynamic task allocation (DTA) and resource balancing and availability (RBA). PTS will arrange the critical jobs based on these conditions of two factors. The proposed approach's core idea is that the task is prioritized based on the criticality of the patient. To begin, the scheduler handles the highest priority tasks, which reflect a patient with high critically. Next, normal tasks are suggested. Each task can have a maximum quantum assigned to it, allowing it to be treated indefinitely. When an agent starts a bargaining process with other agent, the scheduler uses the size indicated by the reference value and the starting agent to calculate the priority once an agent begins a process of negotiation with another agent. In the matrix of reference, task transfers from one agent *i* to another agent (*j*) are designated as *R*_*ij*_.
In Step 2, the agent complete patient task management will be explained. Multi-agent systems will play the role of controlling and scheduling the incoming tasks from PA, and then, FNA will maintain the preprocessing and prediction steps. A personal agent (PA) will run in each gateway. The role of PA is resorting the sensed data through IMoT and migrated with EHR data to generate a new list of tasks and forwarded to fog layer through Wi-Fi and Bluetooth. The another task of PA is checking the resource availability of the connected nodes and then send the stream sensed data to the nearest available node. In each fog node, we have a fog node agent (FNA) that collects the task, a list from PA. After data preprocessing and prediction with diagnosis steps, multi-agent system will assign the tasks according to critically. Patient with sever condition will be assigned to intensive care units (ICU). Patient with moderate condition will be advised to be in continuous monitoring. In last case, when the patient is in mild condition, then they will be advised for further checking. Following are the mathematical presentation of MAA role:
  (6) $$\begin{array}{c} B=\left\{k_{i},\ldots ,k_{n},r_{i},\ldots ,r_{n},w_{i},\ldots ,w_{n},O_{i},\ldots ,O_{n},a_{i},\ldots ,a_{n},h_{i},\ldots h_{n},c_{i},\ldots c_{n},d_{i},\ldots ,d_{n},\mu ,\sigma \right\}, \end{array}$$
where *k*_*i*_, with *i* = 1, *n*, are the tasks; *r*_*i*_, with *i* = 1, *n*, priority of the *i*th task; *w*_*i*_, with *i* = 1, *n*, is the workload for the *i*th task; *O*_*i*_ with *i* = 1, *n* is the PA output size for the *i*th task; *A*_*i*_, with *i* = 1, *n*, is the required accuracy for the *i*th task; *m*_*i*_, with *i* = 1, *n*, is the demanded resources for the *i* task; *h*_*i*_, with *i* = 1, *n*, hashes of tasks; *c*_*i*_, with *i* = 1, *n*, the acceptable maximum cost for each task given by the service demander; *d*_*i*_, with *i* = 1, *n*, delivery location of *i*th task; 1/4 means workload of all scheduled batches in all nodes and cloud.
For every scheduled batch, the standard deviation of load is calculated. The standard deviation and mean 1/4 of the workloads are calculated to consider the current workload to those of previous tasks. As illustrated in equation (7), this allows us to see whether a workload of the tasks is below a specific threshold.
  (7) $$\begin{array}{c} \left|w_{i}\right|<a*y, \end{array}$$
where *α* is an adjustment parameter to be calculated.
In Step 3, all services request (PA) if the workload is over the threshold. This allows for a manner of global optimization to be carried out in order to maintain a specific level of balance in the global sensor network, such as not overloading a node or assigning only minor tasks to a certain node. FNA also is capable of monitoring tasks by checking task attributes like integrity and size of the task in order to execute a specific type of local optimization.
In Step 4, PA will perform task scheduling decision for incoming task processing in current node (in case of the task size fit the local node resources) shifting to neighbour fog nodes (when the current node suffer from lake of resources). Indeed, PA will decide according to a set of features (load balancing, priority, and resource availability). In other words, three main decisions will be produced by PA: execute locally, execute in neighbour, and execute in the cloud. FNA will provide the cost and available resources from cost function, according to the cost and the history of each patient, through patient health record (PHR) from the cloud, tasks are scheduled. See MAA steps below.
In brief, MAA has 4 main steps, starting with collecting the tasks from the connected sensors, sorting the tasks according to their critical condition, calculating the threshold of each fog node, and distributing the tasks among fog nodes depending on the workload.

*(1) Cost Function*. This function's primary job is to compute the cost of processing a task based on available resources and the complexity of the task.

The article "Smart Healthcare System for Severity Prediction and Critical Tasks Management of COVID-19 Patients in IoT-Fog Computing Environments" was retracted in 2023. Reasons: signs of a paper mill; suspected computer-generated content; unreliable results or conclusions; lack of ethics approval or compliance.

Task complexity, local workload (LW), neighbour workload (NW), and cloud workload (CW) will all be included in the cost function.

*(2) Task Processing*. Every agent in each fog node has its own processing unit that has its own set of computation resources. The cost function receives the current workload. (Algorithm 1)

*(3) Collaborative Function*. This function is in charge of the collaboration and interaction among fog node agents in order to share current workload of nodes and tasks.

#### 4.5.2. Deadline-Aware Algorithm (DAA)

However, the MAA responsible for the initial task assignment, the study controls the failure and migration of nodes and tasks handles in Algorithm 2 (DAA) and maintains their execution under deadlines. If the initial schedule tasks missed the deadline or stop processing due to node failure, then scheduler transfers the request or migrates the workload of tasks to another fog node for the further execution. However, if the fog nodes are busy, the workload will migrate to the cloud computing for the further processing until and unless tasks meet their deadlines. To end, scheduler algorithm also has four main steps, starting with verifying all nodes workload taking into account the deadline, migrating the tasks that missed the deadline to another fog node or cloud datacentres to avoid dropping the task, checking the threshold of fog nodes, and processing the tasks by comparing the threshold with the workload to decide either assigning the tasks to local node, neighbour node, or cloud datacentres.

## 5. Results and Discussion

This section analysed the results of the considered SHSSP-CTM of COVID-19 patients in IoT-Fog computing environments via different techniques, whereas widely exploited methods for predicting the severity of COVID-19 data primarily depend on shallow severity prediction and statistical models. The severity prediction that considers combination relationships among different features is proposed to improve prediction accuracy. Therefore, based on different features, the study discusses different result analyses of different methods.

### 5.1. Severity Prediction Results Based on Single Feature Set

The severity prediction has performed mainly on two models such as RF and RL to predict the features of any data based on their attributes. Initially, the study predicts the results of data based on single feature set in order to obtain the performances of different classes such as mild, moderate, and sever. The initial obtained result is shown in Table 2.

The article "Smart Healthcare System for Severity Prediction and Critical Tasks Management of COVID-19 Patients in IoT-Fog Computing Environments" was retracted in 2023. Reasons: signs of a paper mill; suspected computer-generated content; unreliable results or conclusions; lack of ethics approval or compliance.

Table 2 demonstrates the performance result of different schemes based on different features in demographic feature set. However, the results showed that LR model has leading performance in the all evaluation measurements comparing with RF. In the most of metrics, both of the models have shown only small difference in the results, but the big difference can be seen in precision and recall.

Table 3 demonstrates the prediction results based on chronic condition feature set. We have found a small difference in the obtained results in most of classification measurements except F1 and precision where RF outperformed LR with high rate.

Table 4 demonstrates the classification results based on symptom feature set. The introduced classification results indicated that RF outperformed the LR in all evaluation metrics, but the most highest difference results were in precision followed by F1.

Table 5 presented the prediction results for selected classifiers based on laboratory finding feature set. The results demonstrated that RF has leading performance in all of prediction indicators.

Table 6 introduced classification results based on vital sign feature set. According to the achieved results, the most dominant prediction model is LR.

LR has scored a significant performance in all evaluation measurements, especially accuracy and F1. Comparing with RF, LR presented a significant difference in results with value of 16% in both mentioned metrics. To end, in all previous five feature sets, each of RF and LR has provided a varied classification performance. The obtained results can be interpreted into two views. On the one hand, the RF is the best model for the prediction of COVID-19 severity when feature vector based on chronic conditions, symptoms, and laboratory findings. On the other hand, LR is the best COVID-19 severity prediction model for classification task based on features extracted from demographic and vital sign data.

### 5.2. Severity Prediction Results Based on Feature Fusion

The severity prediction model with feature fusion method widely exploited to get the optimal accurate results on the data. The incorporation of several different types of feature information in order to gain more popular feature information is known as feature fusion. Different methods of feature fusion can yield different results. The importance of selecting a suitable fusion method for improving accuracy cannot be overstated. The models such as RF and LR extends used in the COVID-19 dataset to obtain the exact reason of disease. Therefore, severity prediction based on feature fusion implemented in the study as the results displayed in Table 7.

The article "Smart Healthcare System for Severity Prediction and Critical Tasks Management of COVID-19 Patients in IoT-Fog Computing Environments" was retracted in 2023. Reasons: signs of a paper mill; suspected computer-generated content; unreliable results or conclusions; lack of ethics approval or compliance.

Table 7 compared the performances of different schemes based on different component metrics; RF outperformed LR model in all prediction performance measurements except AUC where LR scored 87% and RF scored 83.3%.

### 5.3. Severity Prediction Results Based on Feature Fusion and Selection Method

The severity prediction-based feature fusion and selection technique jointly can achieve optimal results. Each of RF and LR classification with fused feature vector has presented significant prediction accuracy for COVID-19 patients. The importance of selecting a suitable fusion method for improving accuracy cannot be overstated. The suggested methods obtained various results as displayed in Table 8.

Table 8 shows the RF has outperformed LR model with average score reach to 7% in each of accuracy, F1, recall, and precision. On the other hand, LR surpassed the RF with 3% into AUC.

However, the obtained accuracy in each individual set needs to be compared with grouped sets. Therefore, Table 9 shows the overall improvements that obtained when we used the fusion set and fusion set combined with feature selection protocol.

According to Table 9, comparing with average prediction based on five sets (demographic, chronic, symptoms, laboratory, and vital), the accuracy has improved to 18.74% for RF model and 14.88% into LR model based on fusion set. Further improvements have been achieved based on fused and selected features where 7.8% rate scored for RF model and 5.1% for LR model.

A confusion matrix is constructed, which indicates how well a classification model (or “classifier”) implements on a collection of test information for which the true values are recognized. The uncertainty matrix itself is straightforward, yet the related terms can be explained as shown in Figure 3.

The highest classification accuracy for RF model was obtained based on mild and severe data. Where these two classes have outperformed, the moderate with average classification ratio reaches to 15%. This indicates that the performance of RF has less errors based on sever and mild data.

A classification model categorizes data into two or more classes. Detecting one or another class is often needed and costs nothing extra. We might, for example, want to distinguish between white and red wine equally. It may be difficult to differentiate representatives of one disease from that of another.

The article "Smart Healthcare System for Severity Prediction and Critical Tasks Management of COVID-19 Patients in IoT-Fog Computing Environments" was retracted in 2023. Reasons: signs of a paper mill; suspected computer-generated content; unreliable results or conclusions; lack of ethics approval or compliance.

Class distribution is also significant when assessing the efficiency of classification models. When it comes to disease identification, the number of disease carriers can be negligible when compared with the healthy population. The first step in testing every classification model is to test its confusion matrix. Many model statistics and accuracy metrics are created on top of this uncertainty matrix.

As shown in Figure 4, the highest classification accuracy for LR model was obtained based on severe data followed by moderate and mild class subsequently. Where sever class has outperformed, other two classes with average classification ratio reach to 7% compared with moderate and 10% compared with mild class. To mention, the performance of LR classifier has less classification errors based on sever patient data. Also, the RF classifier has low classification errors compared with LR model.

The *x*-axis is FP rate and TP rate as defined aforementioned in table shape. Random forests create complicated determination values by randomly examining FP and TP values and their results to predict the target variable. As a result, random forests outperform LR in terms of precision. Furthermore, when several (types of) explanatory variables are added to a random forest model, random forests can be used to investigate the relationship between explanatory variables and diseases.

In Figure 5, ROC for mild class shows the RF prediction model outperforms as compared to RL in terms of different matrixes to predict features of healthcare dataset. The main reason is that the prediction power of random forest is N rounded with lightweight time iteration as compared to RL during the process of data in the different schemes.

Random forests create complicated determination values by randomly examining FP and TP values and their results to predict the target variable. In both moderate and sever classes, figures as the green lines show the potential strength as compared to pink in terms of accuracy, precision, and recall metrics. Therefore, the lightweight iteration of random forest as compared to RL is optimal for all classes of prediction method as shown in Figure 6 (ROC for moderate class) and Figure 7 (ROC for sever class).

## 6. Resource Management Experimental Results

We use the Java-created simulator (iFogSim) toolkit for simulating the embedded architecture and the environment for illustrating the viability of our suggested cloud-fog model and integration with traditional cloud (T-cloud) solution. We have run the data 5 rounds; in each round, we change the specifications of T-cloud and cloud-fog to show the performance of proposed model. The experimental simulation was carried out on the computer system having 16 GB Ram, 3.2 Processor, Core i5, 6th Gen HP, 500 GB HDD Windows 10 genuine 64-bit Operating System.

The article "Smart Healthcare System for Severity Prediction and Critical Tasks Management of COVID-19 Patients in IoT-Fog Computing Environments" was retracted in 2023. Reasons: signs of a paper mill; suspected computer-generated content; unreliable results or conclusions; lack of ethics approval or compliance.

### 6.1. Resource Usage

In this section, we will show the resource usage management in our proposed model in a comparison with traditional cloud environment.  Figure 8 shows the experimental results.

The resource usage in proposed system indicates the complete resource management overall network. For the first run, we established 2 datacentres in cloud environment; we got 1719 kbps of used resources in T-cloud. For the same amount of data, we establish 4 gateways to forward the sensed data to fog layer, and we got 2546.2 kbps using cloud-fog model.

In the second run, we increased the number of cloud datacentres into 3; we got 2590 kbps using T-cloud. For the same amount of data, we got 8213.6 kbps using cloud-fog model for the same number of gateways.

In the third run, we fixed the number of cloud datacentres into 4; we got 3934 kbps using T-cloud. For the same amount of data, and same number of gateways, we got 10227 kbps using cloud-fog model. For the fourth run, we got 5908 kbps using T-cloud. Whereas, in cloud-fog model, we doubled the number of gateways to 8, we got 12306.4 kbps. In last run, we got 9883 kbps in T-cloud. Whereas, in cloud-fog model, we increased the number of gateways to 12, we got 13364 kbps.

### 6.2. Delay

In this section, we will show the delay management in our proposed model in comparison with traditional cloud environment.  Figure 9 shows the experimental results.

The delay in proposed system indicates the complete resource management overall network. For the first run, we establish 3 datacentres in cloud environment; we got 150.3 ms of delay in T-cloud. For the same amount of data, we established 5 gateways to forward the sensed data to fog layer, and we got 19.015 ms using cloud-fog model. In the second round, we increased the number of cloud datacentres into 5; we got 300.445 ms using T-cloud. For the same amount of data, we increased the number of gateways into 8, and we got 48.365 ms using cloud-fog model. In the third run, we increased the number of cloud datacentres into 7, and we got 403.45 ms using T-cloud. For the same amount of data, we increased the number of gateways into 13, and we got 128.891 ms using cloud-fog model.

In the fourth round, we increased the number of cloud datacentres into 8, and we got 413.9 ms using T-cloud. For the same amount of data, we increased the number of gateways into 15, and we got 132.82 ms using cloud-fog model. In the last round, with same amount of cloud datacentres, we got 523 ms in T-cloud. For the same amount of data, we increased the number of gateways into 16, and we got 139.8 ms using cloud-fog model.

The article "Smart Healthcare System for Severity Prediction and Critical Tasks Management of COVID-19 Patients in IoT-Fog Computing Environments" was retracted in 2023. Reasons: signs of a paper mill; suspected computer-generated content; unreliable results or conclusions; lack of ethics approval or compliance.

## 7. Comparison with State-of-the-Art Methods

Benchmarking is the most basic step that must be employed in most of the medical data and image processing study to decide the reliability and efficiency of the improved approaches in comparison with the current one. Commonly, the benchmarking is accomplished either using a standard dataset or the methods for a similar problem domain.

Therefore, the benchmarking in this study was completed by utilizing the best and most up-to-date methods for COVID-19 classification existing in the literature. This study has included fair comparison with the existing state-of-the-art methods in terms of AUC, accuracy, F1, precision, and recall parameters for the performance of severity prediction.

The comparison results are shown in Table 10 with each class and method. Furthermore, the comparison has presented based on all prediction classes such as mild, moderate, and severe. All state-of-the-art works have been trained and tested based on the same dataset. Reference [7, 20] exploited severity prediction model based on RF, SVM, and LR and NN as well as other methods to obtain the degree of different tuples.

As shown in Table 10, study [7] obtained the results of different dataset benchmarks via different classes of different methods with different metrics. The study [7] obtained accuracy of 70%, 80%, and 50%, and precision of 48.6% during the experiment, while study [20] obtained optimal values as compared to study [7] only in terms of AUC 95%. Comparing with work [20], the proposed work has less AUC results but still near to efficient performance.

However, the proposed work obtained more optimal results as compared to Reference [7, 20] in almost all performance measurements to run the benchmark workloads in the system. However, the proposed model not only reduces the complexity but also improves the accuracy and precision optimization values during experiment with lightweight iteration compared with all baseline studies. Furthermore, by analysing the proposed ML outcome distributions, we can see that it is very close to the actual output distribution of the dataset. Also, comparing with other works, in the proposed work, we can see that LR model takes a high advantage in terms of accuracy from the feature vector that obtained from fusion and feature selection approach. In the same time, RF has great benefits from the proposed feature vector in most of performance metrics. To end, by using the proposed work, clinicians can improve the therapeutic effects and reduce the mortality with more accurate and efficient use of medical resources.

The article "Smart Healthcare System for Severity Prediction and Critical Tasks Management of COVID-19 Patients in IoT-Fog Computing Environments" was retracted in 2023. Reasons: signs of a paper mill; suspected computer-generated content; unreliable results or conclusions; lack of ethics approval or compliance.

## 8. Study Limitations

Like other scientific studies, this study has some constraints and limitations. Two drawbacks need to be addressed shortly, as follows:

- The number of patients' data is relatively small, and more data are required in the future. Therefore, the accuracy of the prediction from a large dataset better shows the algorithm's efficiency than the accuracy of prediction from a midrange or small dataset.
- The selected prediction features need to be examined by different methods and highlight the most critical features from the perspective of different approaches.

## 9. Conclusion

With an insanely broad range of clinical scenarios (from infected individuals to critically ill patients), the exceptionally high level of disease transmission requires extraordinary study attempts focused principally on finding more reliable assessment tools. This research presents a Smart Healthcare System for Severity Prediction and Critical Tasks Management (SHSSP-CTM) for COVID-19 patients. On the one hand, different methodological steps have been proposed to achieve high prediction power for the severity of COVID-19 patients, such as data fusion, data normalization, and feature selection.

LR and RF models have been used as baseline models to evaluate the proposed steps, and then, model with high accuracy was selected as the final COVID-19 severity prediction model. On the other hand, MAA has presented to prioritize the COVID-19 patient and provide an efficient management procedure for IoT-Fog network. Our results indicate that data fusion with feature selection presented a maximum prediction power, and it may be utilized for automated severity valuation of COVID-19. The laboratory finding feature set had the most substantial effect on the performance of model. Comparing with every single set of COVID-19 features, significant improvements in severity prediction have achieved based on proposed fused and selected COVID-19 features. Furthermore, RF model had the highest COVID-19 severity prediction performance compared with state-of-the-art methods. MAA algorithm provided efficient prioritization and scheduling performance.

Efficient resource usage, minor delay, and less energy consumption have been observed using MAA. The proposed system can be used as a decision tool that forecasts the severity of COVID-19 in admitted patients. Also, it potentially aids in triaging patients with COVID-19 and prioritizing care for patients at a higher risk of severe disease. Thus, a critical response by the medical organization can be guaranteed to present. The future work will consider a different combination of COVID-19 features and different machine learning models.

The article "Smart Healthcare System for Severity Prediction and Critical Tasks Management of COVID-19 Patients in IoT-Fog Computing Environments" was retracted in 2023. Reasons: signs of a paper mill; suspected computer-generated content; unreliable results or conclusions; lack of ethics approval or compliance.

## Figures and Tables

**Figure 1:** Smart Healthcare System for Severity Prediction and Critical Tasks Management (SHSSP-CTM) of COVID-19 patients.

**Figure 2:** COVID-19 severity prediction.

**Figure 3:** RF confusion matrix.

**Figure 4:** LR confusion matrix.

**Figure 5:** ROC for mild class.

**Figure 6:** ROC for moderate class.

**Figure 7:** ROC for sever class.

**Figure 8:** Resource usage.

**Figure 9:** Delay.

**Algorithm 1:** MAA steps.

**Algorithm 2:** DAA steps.

**Table 1:** Clinical, laboratory, vital functions, and medical history information collected from hospitals records.

Characteristics	Overall appearance
Age, mean (years)	52.83

*Gender, n (%)*	
Male	46 (58.97%)
Female	32 (41.03%)

*Chronic diseases, n (%)*	
Chronic medical illness (hypertension; diabetes; tumour or any type of cancer)	41 (52.56%)

*Outcomes, n (%)*	
Mortality rate	11 (14.1%)
Survival rate	67 (85.9%)

*Symptoms on onset, n (%)*	
Fever	53 (67.95%)
Cough	46 (58.97%)
Generalized weakness	52 (66.67%)
Nasal congestion	33 (42.30%)
Rhinorrhoea	33 (42.30%)
Sneezing	44 (56.41%)
Sore throat	45 (57.69%)
Pleuritic chest pain	42 (53.84%)
Diarrhoea	41 (52.56%)
Lost sense of smell	71 (91.02%)
Lost sense of taste	72 (92.30%)

*Laboratory test, n: abnormal cases based on WHO test range (%)*	
Haemoglobin (g/dL)	M: 11 (23.91%), F: 15 (46.87%)
White blood cell count	31 (39.74%)
Lymphocyte count	13 (16.66%)
Platelet count	13 (16.66%)
C-reactive protein (mg/L)	48 (61.53%)
Urea (mmol/L)	22 (28.20%)
Creatinine (*µ*mol/L)	56 (71.79%)

*Vital signs, n: abnormal cases based on WHO test range (%)*	
Saturation of oxygen in the blood (SPO_2_), (>90, 90–94, 95–100)	46 (58.97%), 21 (26.93%), 11 (14.10%)

**Table 2:** COVID-19 severity prediction based on demographic feature set.

Model	AUC	Accuracy	F1	Precision	Recall
RF	58	50	49.7	49.6	50
LR	60.9	58.9	52.8	69	58.9

**Table 3:** COVID-19 severity prediction based on chronic condition feature set.

Model	AUC	Accuracy	F1	Precision	Recall
RF	54.8	47.4	39.1	48.6	47.4
LR	54.2	48.7	35	41.5	48.7

**Table 4:** COVID-19 severity prediction based on symptom feature set.

Model	AUC	Accuracy	F1	Precision	Recall
RF	67.6	56.4	54.6	55.7	56.4
LR	56.2	44.8	41.4	40.2	44.8

**Table 5:** COVID-19 severity prediction based on laboratory finding feature set.

Model	AUC	Accuracy	F1	Precision	Recall
RF	88.3	75.6	75.9	76.6	75.6
LR	86.6	73	73	73	73

**Table 6:** COVID-19 severity prediction based on vital sign feature set.

Model	AUC	Accuracy	F1	Precision	Recall
RF	88.3	75.6	75.9	76.6	75.6
LR	86.6	73	73	73	73

**Table 7:** COVID-19 severity prediction depending on feature fusion.

Model	AUC	Accuracy	F1	Precision	Recall
RF	83.3	78.2	77.8	78.5	78.2
LR	87.1	74.3	74.2	74.5	74.3

The article "Smart Healthcare System for Severity Prediction and Critical Tasks Management of COVID-19 Patients in IoT-Fog Computing Environments" was retracted in 2023. Reasons: signs of a paper mill; suspected computer-generated content; unreliable results or conclusions; lack of ethics approval or compliance.

**Table 8:** COVID-19 severity prediction depending on feature fusion and selection protocol.

Model	AUC	Accuracy	F1	Precision	Recall
RF	93	86	85.7	87.2	86
LR	90.3	79.4	79.5	79.6	79.4

**Table 9:** Overall accuracy improvements.

Model	Demographic	Chronic	Symptoms	Laboratory	Vital signs	Average of five sets	Fusion set	Fusion and selection protocol
RF	50	47	56	75	67	59	78	86
LR	58	48	44	73	71	59	74	79

**Table 10:** Comparison of benchmarked studies.

Study	Prediction model	AUC	Accuracy	F1	Precision	Recall
[7]	RF	n/a	70	n/a	n/a	n/a
	SVM	n/a	80	n/a	n/a	n/a
	LR	n/a	50	n/a	n/a	n/a

[20]	NN	78.2	n/a	41.3	48.6	n/a
	LR	**95**	n/a	60.4	76.4	n/a

Our	RF	93	**86**	**85.7**	**87.2**	**86**
	SVM	91	79.4	79.1	81	79.4
	NN	86.4	79.4	79.4	79.7	79.4
	LR	90.3	79.4	79.5	79.6	79.4

## Data Availability

All data used in this research are authorized by Al Aziziya Primary Healthcare Sector/Wasit Health Directorate/Ministry of Health, and there is a letter in this regard. Data can be obtained from the corresponding author upon request.
